# *In Vivo* Clearance of Apoptotic Debris From Tumor Xenografts Exposed to Chemically Modified Tetrac: Is There a Role for Thyroid Hormone Analogues in Efferocytosis?

This article has been retracted.

**DOI:** 10.3389/fendo.2022.745327

**Published:** 2022-03-04

**Authors:** Kavitha Godugu, Shaker A. Mousa, Gennadi V. Glinsky, Hung-Yun Lin, Paul J. Davis

**Affiliations:** ^1^ Pharmaceutical Research Institute, Albany College of Pharmacy and Health Sciences, Rensselaer, NY, United States; ^2^ Institute of Engineering in Medicine, University of California, San Diego, CA, United States; ^3^ Ph.D. Program for Cancer Molecular Biology and Drug Discovery, College of Medical Science and Technology, Taipei Medical University, Taipei, Taiwan; ^4^ Cancer Center, Wan Fang Hospital, Taipei Medical University, Taipei, Taiwan; ^5^ Traditional Herbal Medicine Research Center of Taipei Medical University Hospital, Taipei Medical University, Taipei, Taiwan; ^6^ Department of Medicine, Albany Medical College, Albany, NY, United States

**Keywords:** chemokine, efferocytosis, integrin αvβ3, phagocytosis, tetraiodothyroacetic acid (tetrac)

## Abstract

Apoptosis is induced in cancer cells and tumor xenografts by the thyroid hormone analogue tetraiodothyroacetic acid (tetrac) or chemically modified forms of tetrac. The effect is initiated at a hormone receptor on the extracellular domain of plasma membrane integrin αvβ3. The tumor response to tetrac includes 80% reduction in size of glioblastoma xenograft in two weeks of treatment, with absence of residual apoptotic cancer cell debris; this is consistent with efferocytosis. The molecular basis for efferocytosis linked to tetrac is incompletely understood, but several factors are proposed to play roles. Tetrac-based anticancer agents are pro-apoptotic by multiple intrinsic and extrinsic pathways and differential effects on specific gene expression, e.g., downregulation of the X-linked inhibitor of apoptosis (XIAP) gene and upregulation of pro-apoptotic chemokine gene, CXCL10. Tetrac also enhances transcription of chemokine CXCR4, which is relevant to macrophage function. Tetrac may locally control the conformation of phagocyte plasma membrane integrin αvβ3; this is a cell surface recognition system for apoptotic debris that contains phagocytosis signals. How tetrac may facilitate the catabolism of the engulfed apoptotic cell debris requires additional investigation.

## Introduction

The phagocytotic clearance of apoptotic cells in nonmalignant and malignant tissues is a process designated efferocytosis (1–6). The molecular mechanisms that underlie efferocytosis are incompletely understood (2, 5), but involve signals generated by apoptotic cells that attract and engage macrophages and other cells that can express phagocytic function. We have described a cell surface receptor for thyroid hormone analogues on integrin αvβ3 that is generously expressed by cancer cells (7, 8). At this receptor, hormone analogue tetraiodothyroacetic acid (tetrac) and chemically modified tetrac induce tumor cell apoptosis by multiple mechanisms (8–10). This pharmacologic anticancer activity has been associated in human tumor xenografts with substantial graft shrinkage and disappearance of apoptotic cell debris (11–17). The mechanisms of anticancer activity of thyroid hormone analogue actions on tumor cells have been extensively studied; here we examine these actions for ways in which they may contribute to efferocytosis. Tetrac derivatives are also anti-angiogenic and the clearance of blood vessel debris in angiogenic models has been found to be efficient and is not associated with hemorrhage (18, 19); this is in contrast to certain other anti-angiogenic agents such as antibodies to vascular growth factors (20, 21).

We assume that phagocytosis of apoptotic endothelial cells in tetrac-treated models is *via* one or more mechanisms similar to that in efferocytosis in tumor grafts. Integrin αvβ3 has been implicated in the ‘recognition’ by phagocytosing cells of tumor cells (4, 5), as discussed below. The binding of thyroid hormone analogues by αvβ3 may induce important changes in the conformation of the extracellular component of the integrin (‘activation’) (22). Eighty percent of the protein is extracellular (23, 24). Such conformational changes facilitate the interaction of phagocytes and apoptotic tumor cells and uptake of treatment-damaged cancer cells by phagocytes. Thyroid hormone can facilitate phagocytosis of bacteria by a mechanism that depends on αvβ3 (25). If the apoptosing cancer cell is interacting with platelets, thyroid hormone may induce local release of ATP by the platelet and the ATP may act to facilitate monocyte/phagocyte recognition of the apoptotic cell (5). It is observations such as these that encouraged the current work.

It is important to appreciate that tetrac and the principal product of the thyroid gland–L-thyroxine (T4)–from which tetrac is derived have radically different functions at the thyroid hormone receptor on integrin αvβ3 (8, 10). For example, T4 is anti-apoptotic (9) and thus will not contribute to efferocytosis. In contrast, tetrac and chemically modified versions of tetrac, are pro-apoptotic *via* αvβ3 and block the anti-apoptotic actions of T4 (9). The action described in the current report of tetrac on efferocytosis related to tumor cells undergoing apoptosis is novel, but glucocorticoids (26, 27) and parathyroid hormone (PTH) (28) are examples of other hormones recently shown to modulate efferocytosis linked to wound-healing and clearance of the debris of the inflammatory process.

The clearance by phagocytes of apoptotic cells from a tissue field is widely regarded to involve three processes. These are generation of apoptotic announcement (‘find me’) and pro-phagocytotic (‘eat me’) signals that may be read by appropriate white blood cells and the post-engulfment processing of debris (2, 5).

## Experimental

### Materials and Methods

P-bi-TAT was synthesized at the Pharmaceutical Research Institute (PRI, Rensselaer, NY 12144) (29). Dulbecco’s Modified Eagle’s Medium (DMEM), fetal bovine serum (FBS), penicillin, streptomycin, and trypsin/ethylenediaminetetraacetic acid (EDTA) were purchased from Sigma Aldrich (St. Louis, MO, USA). Human glioblastoma U87-luc cells were purchased from ATCC (Manassas, VA, USA) and human primary cells (GBM 052814) were a generous gift from the University of Pittsburgh Medical Center (Department of Neurosurgery).

### Cell Culture

Human glioblastoma U87-luc and GBM 052814 cells were grown in DMEM that was supplemented with 10% FBS, 1% penicillin, and 1% streptomycin. Cells were cultured at 37°C to subconfluence and treated with 0.25% (w/v) trypsin/EDTA to induce cell release from flasks. Cells were washed with culture medium that was free of phenol red and FBS and counted.

### Animals

Immunodeficient female NCr nude homozygous mice aged 5-6 weeks and weighing 18-20 g were purchased from Taconic Laboratories (Germantown, NY, USA). All animal studies were conducted at the animal facility of the Veteran Affairs (VA) Medical Center, Albany, NY, USA in accordance with current institutional guidelines for humane animal treatment and approved by the VA IACUC. Mice were maintained under specific pathogen-free conditions and housed under controlled conditions of temperature (20-24°C) and humidity (60-70%) and 12 h light/dark cycle. Animals were fed a standard pelleted mouse chow. Mice were allowed to acclimatize for 5 days before study.

### Glioblastoma Xenografts and Treatments

For the glioblastoma tumor model, U87-luc and GBM 052814 were harvested, suspended in 100 μL of DMEM with 50% Matrigel^®^ and 2 × 10^6^ cells were implanted subcutaneously dorsally in each flank, achieving two independent tumors per animal. Immediately prior to initiation of treatments, animals (n=40) were randomized into treatment groups (5 animals/group) by tumor volume measured with Vernier calipers. After detection of a palpable tumor mass (4-5 days post implantation), the treatments of control (PBS) or P-bi-TAT (10 mg/kg body weight) were administered daily, subcutaneously, on the ventral side of the animal, for 21 days (ON Treatment) and in another group of mice treatments were administrated daily for 21 days followed by 21 days discontinuation (ON + OFF Treatment). The tumor volume (width and length) was measured with vernier calipers at 3-day intervals during the ON and ON + OFF studies, and the volumes were calculated using the standard formula W X L^2^/2. Animals were humanely sacrificed, and tumors were collected and fixed in 10% formalin.

### Histopathology

The fixed samples were placed in cassettes and dehydrated, using an automated tissue processor. The processed tissues were embedded in paraffin wax and the blocks trimmed and sectioned to about 5 x 5 x 4 µm size, using a microtome. The tissue sections were mounted on glass slides using a hot plate and subsequently treated in the order of 100%, 90%, and 70% ethanol for 2 min each. Finally, the tissue sections were rinsed with water, stained with Harris’s hematoxylin and eosin (H&E), and examined under a light microscope at lower magnification (4X and 10X) and higher magnification (40X). Efferocytosis was defined by percent of total apoptotic tumor cells (TUNEL-positive cells) exhibiting pyknotic nuclei with dark brown staining and pointed apoptosis.

### TUNEL Assay

Analysis of apoptotic cells in tumor tissue was done with terminal deoxynucleotidyl transferase-mediated dUTP nick-end labeling (TUNEL) staining using an HR-DAB detection kit, according to the manufacturer’s directions (Abcam, Cambridge, MA, USA). TUNEL-positive cells had pyknotic nuclei with dark brown staining and pointed apoptosis. Images of the sections were taken with a light microscope (Leica, Buffalo Grove, IL, USA) at 40X and 100X magnification. The percentage of apoptotic cells was calculated on the basis of control (PBS-treated) samples.

### Immunohistochemistry

Tumor sections were deparaffinized in xylene and rehydrated, followed by antigen retrieval with retrieval buffer (sodium citrate buffer, pH 6.0; Abcam). The peroxidase activity was inhibited by 3% hydrogen peroxide for 10 min and the sections were incubated with 10% normal goat serum (Vector Laboratories, Burlingame, CA, USA) to block the non-specific binding of reagents. Rat anti-mouse CD68 antibody (1:100, Bio-Rad, Hercules, CA, USA) was applied as primary antibody overnight in a moist chamber at 4°C. Goat anti-rat immunoglobulin (1:100, Abcam) was applied as secondary antibody for 2 h at 37°C, followed by streptavidin-HRP for detection. Immunostaining was developed with DAB + NI-Chromogen substrate (Vector Laboratories), followed by counterstaining with methyl green. Tumor tissue was examined under the light microscope at magnification 40X and 100X.

CD68-positive cells were developed for light microscopy with DAB + NI-Chromogen substrate (dark-brown staining). Other cells stained green with methyl green (**Figures 2** and **3**, below). The percentage of CD68-positive cells was calculated based PBS-exposed control samples.

### Statistical Analysis

Statistical analysis was performed with GraphPad Prism software (GraphPad, San Diego, CA). Data are presented as means +/- SD. For comparison between 2 data sets, Student’s t test was used; ANOVA was used in comparisons of 3 or more sets of data. *P <0.05, **P <0.01 and ***P<0.001 indicated statistical significance.

## Results

### Efferocytosis

In a series of reports on the actions of chemically modified forms of tetrac, we have shown that the agents are effective in reducing xenograft size by 80-95% (16, 17, 29, 30). In the current study, a substantial decrease was confirmed in the tumor growth rate of xenografts of U87-luc and GBM 052814 cells in response to tetrac-based P-bi-TAT (**Figure 1**).

**Figure 1:** Glioblastoma xenografts implanted in nude mice using U87-luc and primary glioblastoma cells (GBM 052814). Tumor samples were obtained after 21 days of treatment with subcutaneous injection of either PBS and P-bi-TAT (10 mg/kg body weight) (ON treatment) OR an additional 21 days after discontinuation of treatment (ON + OFF treatment model). **(A, C)** Tumor volumes and Tumor weight (U87-luc) **(B, D)** Tumor volumes and Tumor weight (GBM 052814).Values are expressed as mean ± SD, ***P < 0.0001, **P < 0.001.

Histopathologic examination of the xenografts after 3 weeks of P-bi-TAT therapy in U87-luc glioblastoma cells (**Figure 2**) and in a primary culture of glioblastoma cells (GBM 052814) (**Figure 3**) has revealed evidence of apoptosis as indicated by cell shrinkage, blebbing and nuclear fragmentation (31), in the course of xenograft shrinkage of about 90% (29). These findings are in accordance with our previous results (29).

**Figure 2:** Histopathological evaluation of samples of U87-luc xenografts from nude mice after treatment with P-bi-TAT. Tumor sections were subjected stained to H&E staining, TUNEL assay, and CD68 immunohistochemical staining for each group. Tumor samples were obtained after 21 days of treatment with subcutaneous injection of either PBS and P-bi-TAT (10 mg/kg body weight) (ON treatment) OR an additional 21 days after discontinuation of treatment (ON + OFF treatment model). **(A)** Representative images of H&E staining, TUNEL assay, and CD68 staining are presented. Black arrows indicate apoptotic cells and red arrows indicate macrophages. Scale bar 40 X, insert 100 X. **(B)** Percentage of apoptosis of tumor tissues in control and P-bi-TAT was measured with the TUNEL assay. **(C)** Percentage of CD68 positive cells per view in control and P-bi-TAT. Values are expressed as percentage of mean ± SD, ***P < 0.0001, **P < 0.001.

**Figure 3:** Histopathological evaluation of primary glioblastoma cells (GBM 052814) from tumor tissues excised after treatment of nude mice with P-bi-TAT. Tumor sections were stained for H&E staining, TUNEL assay, and CD68 immunohistochemical staining for each group. Tumor sections were obtained after 21 days of daily subcutaneous injection of PBS and P-bi-TAT (10 mg/kg body weight) (ON treatment) and 21 days after discontinuation of treatment (ON + OFF treatment model). **(A)** Representative images are presented of H&E staining, TUNEL assay, and CD68 staining. Black arrows indicate apoptotic cells and red arrows indicate macrophages. Scale bar 40 X, insert 100 X. **(B)** Percentage of apoptosis of tumor tissues in control and P-bi-TAT measured with the TUNEL assay. **(C)** Percentage of CD68 positive cells per view in control and P-bi-TAT. Values are expressed as percentage of mean ± SD, ***P < 0.0001, *P < 0.01.

As shown in histological and immunological staining in the upper panels and summarized in the lower panels of **Figures 2** and **3**, P-bi-TAT induces apoptosis, consistent with our previous results (15). Indicated graphically in the lower panels (**Figures 2B, C** and **3B, C**), discontinuation of the drug for 3 weeks was associated with prototypic efferocytotic clearance of the apoptotic debris. The histological studies indicated that there was no build-up of macrocytes in the tumor xenografts following drug withdrawal. There was no resumption of residual xenograft growth in tetrac-treated animals.

### Necrosis

A limited degree of necrosis was seen in the two GBM models exposed to P-bi-TAT for 3 weeks. H&E staining of control and P-bi-TAT-treated xenografts was used to estimate extent of tissue necrosis, characterized on light microscopy by large, blurred, red-stained material that contained blue-stained nuclear fragments. Non-necrotic areas were characterized by dark purple-stained living cells. We found 5% and 8-10% necrosis, respectively, in treated U87-luc and GBM 052814 cells.

## Discussion

### Induction of Apoptosis and Effectiveness of the Process

The induction of apoptosis in cancer cells by tetrac or chemically modified tetrac involves multiple intrinsic and extrinsic mechanisms (9, 14, 32). Specific serine phosphorylation of p53 is a critical feature of the intrinsic pathway (**Figure 4**) (9), which has been studied as a biochemical site of competition between T4 and tetrac (32–35). The extrinsic pathway depends on activation of caspases (**Figure 4**). In this regard; thyroid hormone analogues have been shown to affect caspases 2 (9), 3 and 9 (10). Tetrac is pro-apoptotic, but T4, the iodothyronine analogue from which tetraci is derived, is anti-apoptotic (10). As an anti-apoptotic factor, T4 decreases activity of specific caspases, whereas tetrac-based agents include caspase activation among their pro-apoptotic actions (9, 10).

**Figure 4:** Schematic overview of extrinsic and intrinsic apoptosis pathways in the cell and points at which thyroid hormone in these pathways is anti-apoptotic. The pathways converge at the mitochondrion and cause its permeabilization, with release of cytochrome c and consequent apoptosis. Genes or proteins circled in red or green identify loci of differential actions of thyroid hormone on these multiple factors in apoptosis that are discussed in the current work. Red and green colors identify downregulation and upregulation of factors respectively. The Fas receptor by its interaction with Fas ligand activates the extrinsic pathway. An intrinsic pathway activator is DNA damage from different factors such as radiation or chemotherapy. Bcl-2, B cell lymphoma-2; Bcl-xL, Bcl-2-related gene, long form; Bad, Bcl-2/Bcl-xL-associated death domain protein; Bak, Bcl-2 homologus antagonist killer protein; Bax, Bcl-2-associated X protein; IAPs, inhibitors of apoptosis; MCL-1, myeloid leukemia cell-1; XIAP, X-linked inhibitor of apoptosis. Reprinted from Lin HY, Glinsky GV, Mousa SA, Davis PJ. Thyroid hormone and anti-apoptosis in tumor cells. Oncotarget. 2015;6(17):14735-14743 under the terms of the Creative Commons Attribution License.

### Apoptotic Cell Signaling: ‘Find Me’ Signal to Phagocytes

The ‘find me’ signals from apoptotic cells to phagocytes include nucleotides such as ATP and UTP and certain chemokines, such as CX3CL1 (fractalkine), that are released by dying tumor cells (4, 5). Nucleotide synthesis is activated by T4 *via* αvβ3, as this pathway has a substantial and positive effect on tumor cell respiration (36). However, tetrac and chemically modified forms of tetrac—such as P-bi-TAT—block cell respiration by downregulating expression of genes that code for ATP synthases and NADH dehydrogenase. These enzymes are a part of mitochondrial respiration in cancer cells. Thus, the anticancer activity of tetrac is likely to reduce the amounts of ATP and of CX3CL1 (34) available for release as apoptosis progresses. A remaining question is, what are the ‘find me’ signaling molecules in efferocytosis induced by tetrac?

The action of tetrac on chemokine expression is generally downregulation (37), but in contrast, chemokine ligand CXCL10 and receptor CXCR4 mRNAs are found in abundance in tetrac-treated human breast and thyroid cancer cells (37) CXCL10 can serve as an attractant for macrophages and T cells (38, 39), as well as being pro-apoptotic (40). CXCR4 is a human and murine macrophage chemokine receptor, shown to be increased in a model of inflammatory disease (peritonitis) (41). Among its functions is promotion of macrophage egress from inflammation sites and entry into lymphatics. A hallmark feature of the global gene expression changes induced by tetrac-based agents at the integrin is that the downstream effects conform to specific pathways that lead to changes in biologic function. These changes should not be viewed as isolated target gene effects. Ongoing studies of the actions of P-bi-TAT on gene expression in GBM cells are consistent with this concept and reveal, as they have in other types of cancer cells (10, 37), actions on efferocytosis-related genes, including those in signal transduction pathways that modulate pro-apoptotic, anti-inflammatory and anti-proteolytic activities (GV Glinsky: unpublished observations).

### Apoptotic Cell Signaling: ‘Eat Me’ (to Phagocyte)

There is general agreement that the plasma membrane αvβ3 of phagocytes is a sensor for apoptotic cell membrane components that incite phagocytosis (4, 5). Tetrac controls the conformation of this integrin between the activated and non-activated state (22). This important effect will modify the ability of the integrin to recognize and consequently bind potential ligands in the plasma membrane of apoptotic tumor cells. In this regard, a number of such ligands have been identified (4, 5). We suspect that a variety of growth factor receptors found on the surface of cancer cells and that communicate with αvβ3 (10) may also be part of the ‘eat me’ paradigm. The chemokine ligand CX3CL1 (fractalkine) may be a component of phagocyte recruitment (3, 42). We would point out, however, that tetrac-based drugs inhibit the expression of a number of chemokines, including fractalkine in cancer cells (9). It would thus seem unlikely for such agents (chemokines) to be present in excess in tumor cells undergoing tetrac-induced apoptosis.

We would also propose that the apoptosis process itself is potentiated by the actions of tetrac molecules to downregulate expression of genes such as the X-linked inhibitor of apoptosis (XIAP) and to upregulate transcription of pro-apoptotic genes such as those for certain caspases (13, 43, 44).

While the clearance of apoptotic tumor cell debris in response to tetrac has been satisfactorily demonstrated, the possibility that tetrac may interfere with phagocytosis of bacteria, e.g., meningococcus, has been raised (25). However, the tetrac effect in this example was demonstrated only in the presence of supraphysiologic concentrations of T4 and T3 and it is not clear whether there is an effect of tetrac or modified tetrac on bacterial clearance when T4 and T3 levels are normal range.

When phosphatidylserine (PtdSer) moves from the inner to the outer plasma membrane leaflet in the early course of apoptosis in cancer cells, it is an ‘eat me’ signal (5). We assume that tetrac-induced apoptosis is associated with PtdSer signaling, however, this process has not yet been verified in tetrac-treated cells.

### Post-Engulfment Phagocyte Handling of Apoptotic Cell and Orientation for Tissue Departure

The migration of phagocytic cells to and from a tissue region of apoptotic cells is in part a function of ‘find me’ signaling, but the rate of migration of phagocytes is at least in part a process regulated by extracellular matrix protein cues. The effect of the cues can be a function of the presence of thyroid hormone analogues. We have shown that extracellular matrix proteins may influence the rate of migration of endothelial cells when thyroid hormone as T4 is present (17). Tetrac blocks this motility rate enhancement action of T4. This effect needs to be examined in phagocytes, since a slowing egress of such cells may facilitate completeness of local phagocytic uptake of debris.

## Conclusions

The anticancer activity of tetrac and chemically modified tetrac in preclinical studies is associated with extensive tumor cell apoptosis and with frank xenograft shrinkage and no local accumulation of cellular debris. These results presented in **Figures 2** and **3** are very satisfactory examples of efferocytosis. As noted above, the extensive literature of efferocytosis is based on signaling that attracts phagocytes to sites of apoptosis and on signaling that activates phagocytes and their capacity to cope with the internalized remnants of dead cancer cells. In the case of tetrac, drug-induced apoptosis is extensive in mechanism, involving multiple intrinsic and extrinsic apoptotic pathways (9). We can assume, then, that the ‘find me’ and ‘eat me’ signals identified in a substantial number of reports are ample in tetrac-treated cancer cells that are undergoing apoptosis. However, except for nucleotides and chemokines, these signaling molecules have not been specifically sought in tetrac-induced apoptotic cells. Further, tetrac has been shown to decrease transcription of a variety of chemokines and we do not know whether genes such as that for CX3CL1 can be expressed in tetrac-exposed cells.

The shrinkage of tetrac-exposed xenografts testifies to the extent of ‘eat me’ signaling from dying cancer cells. The multiple functions of the thyroid hormone analogue receptor on the extracellular domain of αvβ3 suggest that there are changes in the conformation and functions of this integrin (8, 10) that play the major role in the activation of phagocytosis-capable cells that have been attracted to the tumor that is dying. Are the interactions of phagocyte αvβ3 with apoptotic cell bleb proteins–for example, growth factor receptor proteins–’eat me’ signals?

The absence of tumor cell debris in xenografts exposed to tetrac-based agents indicates that the process of ‘engulfment’ must proceed efficiently in phagocytes exposed to tetrac. This issue has not been specifically examined in any model. We raise the possibility that phagocytes activated in the presence of tetrac and apoptotic tumor cells may not only metabolize the internalized cancer cell debris, but also serve to export the tumor tissue debris; this reflects CXCR4-promoted egress from tumor mass of macrophage containing such debris. We know that cell migration in response to extracellular matrix protein cues may be regulated through thyroid hormone actions at αvβ3 (18). However, the initial observations of this phenomenon showed that T4 enhances the effects of cue proteins and tetrac decrease this effect.

Studies are needed to further define the signaling mechanisms activated by tetrac and chemically modified tetrac to advertise the apoptotic process and to stimulate phagocytosis by nearby macrophages.

P-bi-TAT is a chemically-modified thyroid hormone analogue that may be added to glucocorticoids (26, 27) and PTH (28) as a group of hormones that can stimulate phagocytosis and efferocytosis.

## Author’s Note

Portions of this manuscript were presented in a poster by KG, H-YL, SM and PD at the ENDO 2021 conference (March 23-25, 2021), Poster Abstract 8665.

## Data Availability Statement

The raw data supporting the conclusions of this article will be made available by the authors, without undue reservation.

## Ethics Statement

All animal studies were conducted at the animal facility of the Veteran Affairs (VA) Medical Center, Albany, NY, USA in accordance with current institutional guidelines for humane animal treatment and approved by the VA IACUC.

## Author Contributions

PD: conception, drafting the work, and analysis of data. KG: acquisition and interpretation of data for the work. H-YL: analysis and interpretation of data. SM: interpretation of data. All authors contributed to the article and approved the submitted version.

## Funding

The authors declare that this study received funding from NanoPharmaceuticals LLC, Rensselaer, NY, USA. The funder was not involved in the study design, collection/analysis/interpretation of data, the writing of this article or the decision to submit it for publication.

## Conflict of Interest

PD and SM hold stock in a small pharmaceutical company, NanoPharmaceuticals LLC, that is developing anticancer drugs. PD is Chief Scientific Officer at the company.

The remaining authors declare that the research was conducted in the absence of any commercial or financial relationships that could be construed as a potential conflict of interest.

## Publisher’s Note

All claims expressed in this article are solely those of the authors and do not necessarily represent those of their affiliated organizations, or those of the publisher, the editors and the reviewers. Any product that may be evaluated in this article, or claim that may be made by its manufacturer, is not guaranteed or endorsed by the publisher.
